The article "Complex Destabilization in the Mitochondrial Chaperonin Hsp60 Leads to Disease" was published in 2020. Journal: Front Mol Biosci.

# Complex Destabilization in the Mitochondrial Chaperonin Hsp60 Leads to Disease

**DOI:** 10.3389/fmolb.2020.00159

**Published:** 2020-07-14

**Authors:** Alejandro Rodriguez, Daniel Von Salzen, Bianka A. Holguin, Ricardo A. Bernal

**Affiliations:** Department of Chemistry and Biochemistry, The University of Texas at El Paso, El Paso, TX, United States

**Keywords:** chaperonin, GroEL, mtHsp60, chaperonopathy, protein folding

## Abstract

Several neurological disorders have been linked to mutations in chaperonin genes and more specifically to the HSPD1 gene. In humans, HSPD1 encodes the mitochondrial Heat Shock Protein 60 (mtHsp60) chaperonin, which carries out essential protein folding reactions that help maintain mitochondrial and cellular homeostasis. It functions as a macromolecular complex that provides client proteins an environment that favors proper folding in an ATP-dependent manner. It has been established that mtHsp60 plays a crucial role in the proper folding of mitochondrial proteins involved in ATP producing pathways. Recently, various single-point mutations in the mtHsp60 encoding gene have been directly linked to neuropathies and paraplegias. Individuals who harbor mtHsp60 mutations that negatively impact its folding ability display phenotypes with highly compromised muscle and neuron cells. Carriers of these mutations usually develop neuropathies and paraplegias at different stages of their lives mainly characterized by leg stiffness and weakness as well as degeneration of spinal cord nerves. These phenotypes are likely due to hindered energy producing pathways involved in cellular respiration resulting in ATP deprived cells. Although the complete protein folding mechanism of mtHsp60 is not well understood, recent work suggests that several of these mutations act by destabilizing the oligomeric stability of mtHsp60. Here, we discuss recent studies that highlight key aspects of the mtHsp60 mechanism with a focus on some of the known disease-causing point mutations, D29G and V98I, and their effect on the protein folding reaction cycle.

## Introduction

Protein folding is an important aspect of cellular function and viability because the accumulation of misfolded proteins leads to the formation of insoluble aggregates that ultimately cause cell death. Chaperonins form macromolecular protein complexes that assist the proper folding of nascent proteins to obtain the native state and to refold misfolded proteins to prevent aggregation. Absence of chaperonins in cells results in cell death as demonstrated in bacterial, yeast, and mouse models (Cheng et al., 1989; Fayet et al., 1989; Horwich et al., 1993; Fang and Cheng, 2002; Fan et al., 2020). In humans, mitochondrial Heat Shock Protein 60 (mtHsp60) is in charge of folding mitochondrial proteins along with its co-chaperonin Hsp10 (Lubben et al., 1990; Hartman et al., 1992). The mtHsp60 encoding gene *HSPD1* is a nuclear gene that is translated in the cytosol and imported into the mitochondria due to the presence of an N-terminal mitochondrial targeting sequence that is cleaved upon translocation across the mitochondrial membrane (Cheng et al., 1989, 1990; Reading et al., 1989; Singh et al., 1990). A small fraction of Hsp60 resides in the cytosol and also at the cell surface but the function outside of the mitochondria has not been well established (Soltys and Radhey, 1997; Chun et al., 2010; Choi et al., 2015; Kalderon et al., 2015). Chaperonins carry out protein folding cycles in an ATP-dependent manner. ATP binding, hydrolysis, and ADP release prompt conformational changes that drive the catalytic folding cycles (Fayet et al., 1989; Ostermann et al., 1989; Saibil et al., 1993; Levy-Rimler et al., 2001; Fenton and Horwich, 2008; Illingworth et al., 2015). Due to the intrinsic instability of mtHsp60 complexes *in vitro*, much of what is known about mtHsp60 has come from comparing it to mutant versions of its bacterial counterpart GroEL. GroEL exists mainly as a double ring tetradecameric complex with each ring containing a barrel-like central cavity that accommodates substrates and provides a thermodynamically favorable protein folding environment (Viitanen et al., 1992; Horwich et al., 1993; Braig et al., 1994; Xu and Sigler, 1998; Fenton and Horwich, 2008; Hayer-Hartl et al., 2016). However, contrary to the GroEL mechanism, recent structural studies have determined that mtHsp60 in its catalytically active form exists as a single ring (heptamer) or a double ring (tetradecamer). These single ring intermediates have not been well documented in the GroEL folding cycle and require additional studies (Viitanen et al., 1992, 1998; Nielsen and Cowan, 1998; Nielsen et al., 1999; Levy-Rimler et al., 2001; Sun et al., 2003; Chen et al., 2006; Liu et al., 2009; Illingworth et al., 2011; Nisemblat et al., 2014, 2015; Vilasi et al., 2014; Enriquez et al., 2017; Jebara et al., 2017; Bhatt et al., 2018; Yan et al., 2018). Nucleotide binding and release control the association or dissociation of the heptameric rings along their equatorial domains as protein folding takes place inside the mtHsp60 cavity. It is believed that changes in nucleotide affinity or nucleotide-bound complex stability significantly compromise the catalytic activity of mtHsp60 (Ostermann et al., 1989; Saibil et al., 1993; O’Brien and McKay, 1995; Wilbanks and McKay, 1995; Levy-Rimler et al., 2001; Illingworth et al., 2015). Here, we will focus on two HSPD1 point mutations that have been linked to separate neurodegenerative disorders. The mtHsp60 D29G and V98I missense mutations have shown direct correlation to hereditary spastic paraplegia type 13 (SPG13) and mitochondrial Hsp60 chaperonopathy (MitCHAP-60). It has been found that these point mutations act by destabilizing the oligomeric mtHsp60 complex thereby hindering its ability to fold client proteins. It is hypothesized that these loss-of-function mutants pose a high risk of cell damage due to a higher susceptibility to protein aggregate formation. Additionally, there is an inability to fold key proteins involved in the energetic pathways found in mitochondria, the latter resulting in energy deprived cells (Parnas et al., 2009; Wang et al., 2019).

The article "Complex Destabilization in the Mitochondrial Chaperonin Hsp60 Leads to Disease" was published in 2020. Journal: Front Mol Biosci.

## The Chaperonin Protein Folding Cycle

The bacterial homolog of mtHsp60, GroEL, remains the most widely studied of the chaperonins. It is remarkably stable even after chromatography purification and it retains folding activity *in vitro* (Braig et al., 1994; Xu and Sigler, 1998). It is composed of two heptameric rings with their equatorial domains stacked against each other, forming a large double-barrel complex. The architecture of the monomeric protein is constituted of apical, intermediate, and equatorial domains. The apical domain contributes to the formation of the ring opening where substrate is thought to interact, bind, and enter the inner cavity, while the equatorial domain is involved in nucleotide binding and intra-ring communication. The intermediate domain mostly undergoes conformational changes in response to nucleotide binding and dissociation, driving most of the activity inside of the barrel (Horwich et al., 1993; Braig et al., 1994; Xu and Sigler, 1998; Fenton and Horwich, 2008; Hayer-Hartl et al., 2016). GroEL requires the activity of a co-chaperonin, GroES, much like mtHsp60 requires Hsp10 during its own folding cycle (Fayet et al., 1989; Horwich et al., 1993; Weissman et al., 1995; Xu and Sigler, 1998; Hayer-Hartl et al., 2016). GroEL is thought to interact with misfolded substrates via hydrophobic patches near the apical domain and along the inner walls of the barrel. Selectivity for misfolded substrates arises from the exposed hydrophobic patches that are characteristic of partially denatured proteins (Houry, 2001; Horwich et al., 2009). Once inside of the cavity, the substrate is trapped by the binding of GroES to the apical domain of the GroEL barrel. Catalysis is driven by the hydrolysis of ATP that is bound to each GroEL subunit in an ATP binding pocket near the equatorial domain of the complex. Hydrolysis of ATP and subsequent release of ADP trigger conformational changes that induce the folding of the substrate inside the cavity followed by release of GroES and finally the liberation of the folded substrate (Saibil et al., 1993; Weissman et al., 1995; Xu and Sigler, 1998; Fenton and Horwich, 2008; Hayer-Hartl et al., 2016). This folding mechanism is highly controlled and can be seen in other chaperonins such as mtHsp60 albeit with some key differences.

The article "Complex Destabilization in the Mitochondrial Chaperonin Hsp60 Leads to Disease" was published in 2020. Journal: Front Mol Biosci.

MtHsp60 can alternate between single and double heptameric ring conformations upon nucleotide binding and following hydrolysis (Viitanen et al., 1992, 1998; Nielsen and Cowan, 1998; Nielsen et al., 1999; Levy-Rimler et al., 2001; Nisemblat et al., 2014, 2015; Vilasi et al., 2014, 2018; Enriquez et al., 2017; Jebara et al., 2017; Bhatt et al., 2018; Wang et al., 2019; Gomez-Llorente et al., 2020). Furthermore, the structure of the ATP bound conformation has recently been solved, both by crystallography and electron microscopy. In these structures, mtHsp60 adopts a symmetric “American football” like conformation, with two rings sitting against each other via contacts in their equatorial domains, while both rings are capped by one heptameric ring of Hsp10 positioned directly on the apical domain (Nisemblat et al., 2014, 2015; Wang et al., 2019; Gomez-Llorente et al., 2020). Recently, ADP bound mtHsp60 has been shown to separate into single rings capped with an Hsp10 heptamer (Wang et al., 2019). Additionally, nucleotide free mtHsp60 has been shown to form single ring toroidal complexes when reconstituted *in vitro* (Viitanen et al., 1998). It has also been demonstrated, however, that tetradecameric complexes composed of two rings sitting against each other can also be purified intact from bacteria (Enriquez et al., 2017). Although higher resolution structural data are needed to fully support the existing oligomeric state hypotheses, when compared with GroEL, mtHsp60 has unique conformations that are likely important in its folding cycle. Other chaperonins displaying single ring intermediates have also been studied such as the ΦEL chaperonin and the OBP chaperonin, both from bacteriophages. For example, ΦEL exists as a double ring tetradecamer in its nucleotide free and ATP bound states but dissociates into two single heptameric rings in its ADP bound state. The single ring conformation observed in these chaperonins is thought to be a key intermediate in the protein folding cycle and not an off-pathway artifact (Cornelissen et al., 2012; Hildenbrand and Bernal, 2012; Kurochkina et al., 2012; Semenyuk et al., 2015, 2016; Molugu et al., 2016; Bhatt et al., 2018).

It is important to distinguish GroEL and Hsp60, both considered group I chaperonins, from their group II counterparts. Some examples of group II chaperonins include the archaeal thermosome and the eukaryotic TRiC chaperonin. These chaperonins typically vary in subunit number and in some cases, their hetero-oligomeric nature. The archaeal thermosome found in Thermoplasma *acidophilum* consists of stacked eight membered rings with alternating alpha and beta subunits. The eukaryotic TRiC chaperonin, on the other hand, is comprised of eight different subunits forming each ring. Interestingly, these two chaperonins display a significant level of homology in their subunits despite the fact of several different subunits being involved. Another key difference is the absence of a co-chaperonin in group II chaperonins (Trent et al., 1991; Frydman et al., 1992; Phipps et al., 1993; Klumpp et al., 1997; Ditzel et al., 1998; Cong et al., 2012; Lopez et al., 2015). Instead, a “built-in” lid is formed from apical helix protrusions that close the ring opening, trapping substrate in the main cavity. In humans, mutations in the epsilon subunit of TRiC have been linked to neuropathies, analogous to the neuropathies seen in patients with mutations in the Hsp60 encoding *HSPD1* gene (Bouhouche, 2005). In yeast, it was found that introducing similar mutations in conserved regions of the eight different subunits of TRiC results in eight different phenotypes, highlighting the individual significance of each subunit (Amit et al., 2010).

The article "Complex Destabilization in the Mitochondrial Chaperonin Hsp60 Leads to Disease" was published in 2020. Journal: Front Mol Biosci.

Structural and mechanistic diversity is clearly highlighted when comparing chaperonins across various types of organisms. However, one similarity of special importance among chaperonins is the universal dependence on ATP not only as an energy source but as a conformational trigger of the protein folding cycle. ATP binding, hydrolysis, and ADP release are key factors in the folding cycle progression, and disruption of these events have been shown to be deleterious for protein function and cell viability.

## Chaperonopathies and the Role of mtHsp60 in Disease

Chaperonins are ubiquitously expressed across all types of organisms, from bacteriophages to humans (Perezgasga et al., 1999; Hansen et al., 2003; Reissmann et al., 2007; Cornelissen et al., 2012; Kurochkina et al., 2012; An et al., 2017; Fan et al., 2020). They are indispensable for cellular viability because their absence results in cell death. GroEL knockout bacterial strains are unable to grow, even at lower temperatures. This shows that they are not only necessary during stress conditions such as heat shock but also for normal growth (Fayet et al., 1989). Furthermore, it has been found that human mtHsp60/Hsp10 can replace bacterial GroEL/GroES *in vivo* even though it is believed they are mechanistically distinct and demonstrate the universality of their function (Nielsen et al., 1999; Bross and Fernandez-Guerra, 2016). Comparable loss-of-function experiments have been done in yeast with similar results (Fang and Cheng, 2002). In that work, the number of amino acids removed from the c-terminus resulted in a direct effect on cell survival as the removal of 26 amino acids resulted in viable cells at lower temperatures but the removal of 27 amino acids yielded no cell growth. This suggests that the 26 amino acid truncation in Hsp60 resulted in partially functional proteins able to support cell growth. The lack of growth observed after removing just one more amino acid highlights a defined boundary between functional and non-functional Hsp60 and its direct effect on cell survival (Fang and Cheng, 2002). Drosophila survival has also been shown to be dependent on Hsp60 availability (Perezgasga et al., 1999). Additionally, *in vivo* studies have demonstrated that Hsp60 is essential for the survival of mouse embryos. Furthermore, the deletion of Hsp60 in adult mouse cardiomyocytes leads to heart failure and significantly perturbs mitochondrial protein homeostasis and mitochondrial function (Christensen et al., 2010; Fan et al., 2020).

The article "Complex Destabilization in the Mitochondrial Chaperonin Hsp60 Leads to Disease" was published in 2020. Journal: Front Mol Biosci.

While Hsp60 is predominantly found in the mitochondria, during cellular stress, it can be overexpressed and translocated into the cytosol as well as the extracellular space where it has been found to have various moonlighting functions (Henderson et al., 2013). A study has shown that Hsp60 that has yet to have its mitochondrial targeting sequence cleaved is able to oligomerize outside of the mitochondria; however, it is not quite certain whether Hsp60 that gets translocated outside of the mitochondria functions as an oligomer or a monomer (Vilasi et al., 2014). Inside the cytosol, Hsp60 can modulate the yeast proteasome by interacting with various substrates and preventing their degradation, reducing 20S peptidase activity, and increasing protein ubiquitination (Kalderon et al., 2015). Hsp60 can also interact with the IKK complex promoting the phosphorylation-dependent activation of the IKK/NF-κB survival pathway in response to TNF-a (Chun et al., 2010). NF-κB is an important transcription factor for not only the immune system, but also many survival processes. Hsp60 activation of the IKK/NF-κB pathway for survival can be seen in vascular smooth muscle cells where it can prevent apoptosis as well as promote neointimal thickening of the damaged vessels. However, persistent activation of the pathway has been linked to various chronic inflammatory diseases such as cancer and atherosclerosis (Choi et al., 2015). From the cytosol, Hsp60 can leave the inside of the cell and attach itself to the cell’s surface or enter the extracellular space through secretory vesicles (Campanella et al., 2012). Once outside the cell, Hsp60 can stimulate both the innate as well as the adaptive immune system. High amounts of Hsp60 can be found on the cell surface in response to risk factors associated with atherosclerosis and are highly reactive to T-cells (Grundtman et al., 2011). Hsp60 can also activate the ERK/MAPK pathway as well as TLR4 which can induce vascular smooth muscle cell migration, a key contributor to atherosclerosis (Zhao et al., 2015).

The article "Complex Destabilization in the Mitochondrial Chaperonin Hsp60 Leads to Disease" was published in 2020. Journal: Front Mol Biosci.

Chaperonopathies refer to any pathology resulting from a mutated or otherwise altered chaperone. Genetic chaperonopathies include but are not limited to diseases caused by point mutations in the mtHsp60 encoding HSPD1 gene, as well as other pathologies involving different chaperones (e.g., Hsp40) or chaperonins (e.g., TRiC chaperonin). Acquired chaperonopathies are due to non-genetic chaperone defects such as defective post-translational modifications or mis regulated gene expression (Macario, 2007; Lupo et al., 2016). A few examples of known chaperonopathies include dominant distal myopathy (Hsp40), hypomyelinating distrophy (Hsp60), Charcot-Marie-Tooth disease (Hsp27), and Bardet–Biedl syndrome (BBS proteins) (Lupo et al., 2016; Álvarez-Satta et al., 2017; Palmio et al., 2020; Sarparanta et al., 2020). The mtHsp60 gene has been localized to chromosome 2 in humans. The gene for the co-chaperonin Hsp10 is localized in a head-to-head position with respect to Hsp60 (Hansen et al., 2003). Several genetic mutations in the HSPD1 gene have been associated to human disease. These include SPG13 and MitCHAP-60, both neurodegenerative diseases with different symptoms and modes of inheritance (Bross et al., 2007; Cappello et al., 2014; Bross and Fernandez-Guerra, 2016). The first disease-causing mutation associated with mtHsp60 is V98I. This mutation results in an autosomal dominant form of hereditary spastic paraplegia (SPG) linked to SPG13. SPG symptoms are leg stiffness (spasticity) and weakness although their progression can vary depending on the age of onset of the disease. Degeneration of spinal cord nerves is also a characteristic feature of SPGs. It is hypothesized that the genetic dominance of SPG13 is due to the deleterious effect that mutant mtHsp60 has on wild-type mtHsp60. The V98I mtHsp60 mutation compromises the integrity and function of wild-type mtHsp60 protein complexes. It was found that Gro-EL knockout bacteria remained viable if expression of wild-type mtHsp60 was induced. However, mutant mtHsp60 (V98I) was unable to support bacterial cell growth which highlights the effect of the V98I mutation on mtHsp60 function (Hansen et al., 2002, 2007; Fink, 2003; Bross et al., 2008).

The article "Complex Destabilization in the Mitochondrial Chaperonin Hsp60 Leads to Disease" was published in 2020. Journal: Front Mol Biosci.

Unlike SPG13, MitCHAP-60 is an autosomal-recessive disease best described as a hypomyelinating leukodystrophy caused by the D29G missense mutation (Magen et al., 2008). Although MitCHAP-60 is fundamentally like SPG13, major differences characterize the former. MitCHAP-60 is an early onset disease that is better described as a lethal hypomyelinating neurodegenerative disorder. SPG13 is best categorized as a pure SPG if we consider that “pure” SPGs are characterized solely by lower extremity spasticity. However, MitCHAP-60 can be viewed as a “complicated” SPG since it is accompanied by other more severe symptoms (Fink, 2003; Salinas et al., 2008). Additionally, it was found that the D29G mutant is also unable to support the growth of GroEL knockout bacteria although it was not established if the mtHsp60 loss of function was due to a mechanistically similar cause in the two variants (Magen et al., 2008).

Recently, mtHsp60 studies have highlighted some of the effects of the D29G and V98I missense mutations *in vitro* and *in vivo*. Independent groups have shown that both mutations are unable to support bacterial growth in GroEL knockout complementation assays. Furthermore, using malate-dehydrogenase refolding assays, it has been demonstrated that the ATPase activity of both mutant variants is substantially compromised *in vitro* when compared to wild-type mtHsp60. Additional refolding assays have been done using the ATP synthase F1 β-subunit where it was found that the D29G and V98I mutants result in impaired ATPase activity (Wang et al., 2019). It has also been shown that the D29G mutation affects the oligomeric state of mtHsp60. In these studies, at low protein concentrations, mutant mtHsp60 completely dissociated into monomers while wild-type mtHsp60 remained mostly in its oligomeric form (Parnas et al., 2009). Structural studies on both mutants have highlighted the strong effect nucleotide binding has on the mutant mtHsp60 proteins. Electron microscopy and dynamic light scattering studies showed that mtHsp60 harboring either the D29G or V98I mutation dissociated into monomers upon the addition of nucleotide (ATP and ADP had the same effect on complex disruption) (Wang et al., 2019). The nucleotide free (APO) state was able to oligomerize and was stable under experimental conditions suggesting that the mutations have deleterious structural effects mainly during nucleotide binding and or hydrolysis. Interestingly, from the wild-type ATP-bound “American football” structure, it can be observed that both mutations reside in the equatorial domain of mtHsp60 in very close proximity to the nucleotide binding pocket (Nisemblat et al., 2015). This may further substantiate the hypothesis that the mutants are compromised at or near the nucleotide binding domain, prompting oligomer dissociation.

The article "Complex Destabilization in the Mitochondrial Chaperonin Hsp60 Leads to Disease" was published in 2020. Journal: Front Mol Biosci.

## Conclusion and Perspective

In summary, mtHsp60 is an indispensable chaperonin responsible for regulating mitochondrial protein homeostasis and mitochondrial function. Additional moonlighting roles, especially for cytosolic Hsp60, have been suggested to be important across many tissues and organs, but further work is required in order to establish which oligomeric state is responsible for its function. Presence or absence of Hsp60 is now thought to be a significant biomarker for several diseases (Soltys and Radhey, 1997; Chun et al., 2010; Ghosh et al., 2010; Henderson et al., 2013; Choi et al., 2015; Kalderon et al., 2015). MtHsp60 has been shown to successfully replace GroEL in bacteria and support normal cellular growth, highlighting a fundamental functional similarity. However, studies suggest that the two chaperonin systems follow significantly different mechanisms, perhaps best exemplified by the single ring intermediate observed in mtHsp60. Two missense mutations in the mtHsp60 encoding gene *HSPD1* have been linked to the neurodegenerative diseases SPG13 and MitCHAP-60. Recently, *in vitro* studies have shown that mtHsp60 complex stability is affected by these mutations. Low protein concentrations and nucleotide binding resulted in complete oligomer dissociation when compared to wild-type mtHsp60.

Although current research has elucidated some of the effects of these disease-causing mutations, further studies are needed to fully understand the effect of the mutations at a molecular level. High-resolution structural data of mtHsp60 complexes and intermediates are currently limited to the ATP “American football” conformation. It is imperative to have similar data of the ADP and nucleotide-free intermediates to be able to better understand the complete protein folding mechanism of wild-type mtHsp60. Structural information of stable D29G and V98I oligomers would then facilitate the comparison of these to their wild-type counterpart. Furthermore, current structures rely on mtHsp60 mutants that increase complex stability as well as non-hydrolyzable ATP analogs, both of which may produce off pathway intermediates. Studies using wild-type mtHsp60 as well as natural nucleotides may be necessary to obtain a more reliable model of its protein folding cycle.

## Author Contributions

AR and RB contributed to the conception and preparation of the manuscript. AR, RB, DV, and BH contributed to the editing of the manuscript at all points of the preparation process. All authors contributed to the article and approved the submitted version.

The article "Complex Destabilization in the Mitochondrial Chaperonin Hsp60 Leads to Disease" was published in 2020. Journal: Front Mol Biosci.

## Conflict of Interest

The authors declare that the research was conducted in the absence of any commercial or financial relationships that could be construed as a potential conflict of interest.
